# The Role of Jinhuang Powder to Prevent Adverse Effects of Subcutaneous Injection of Enoxaparin Sodium

**DOI:** 10.1155/2022/7806659

**Published:** 2022-08-24

**Authors:** Meng Zhang, Xiang Zhang, Chunlan Wang, Yangfang Shen, Jianan Fu

**Affiliations:** ^1^Department of Gynecological Radiation Oncology, The Cancer Hospital of the University of Chinese Academy of Sciences (Zhejiang Cancer Hospital), Hangzhou, China; ^2^Institute of Basic Medicine and Cancer (IBMC), Chinese Academy of Sciences, Hangzhou, China

## Abstract

**Objective:**

To determine the role of Jinhuang Powder to prevent adverse effects of subcutaneous injection of enoxaparin sodium.

**Methods:**

The clinical data of 97 patients with cervical cancer who were treated with subcutaneous injection of enoxaparin through the lower margin of the deltoid muscle of the upper arm in Zhejiang Tumor Hospital from August 2020 to August 2021 were retrospectively analyzed. All patients were divided into the control group (*n* = 39) and the research group (*n* = 58) according to the different use time periods of Jinhuang Powder. The research group was treated with Jinhuang Powder and enoxaparin sodium at the same time. The control group started to use Jinhuang Powder after the adverse reactions occurred. The induration, subcutaneous bleeding events, and pain were statistically analyzed.

**Results:**

The incidence of induration (3.4% vs 15.4%, *P*=0.036) and subcutaneous hemorrhage (37.9% vs 76.9%, *P*=0.003) in the research group was significantly lower than that in the control group. The pain in the research group was lighter than that in the control group (grade 0–4 pain: 70% vs 28.2%, 19% vs 30.8%, 8.6% vs 23.1%, 1.7% vs 12.8%, 1.7% vs 5.1%, *P*=0.001).

**Conclusion:**

Preventive use of Jinhuang Powder can significantly reduce the incidence of subcutaneous induration and subcutaneous bleeding and can effectively alleviate the local pain of injection. It is worthy of further study to clarify its role and mechanism.

## 1. Introduction

Cervical cancer is the fourth most common type of cancer in women after breast, colorectal, and lung cancer, and it is also the fourth most common cause of cancer death in women. The International Agency for Research on Cancer (IARC) estimated that more than 600,000 women worldwide were diagnosed with cervical cancer in 2020, and about 340,000 women died from the disease. The literature has shown that the incidence of deep vein thrombosis (VTE) in cervical cancer patients is as high as 41.5% [1]. In addition to increasing the mortality rate of patients, VTE will interfere with patient care plans and treatment plans and will also reduce the quality of life of patients. Therefore, anticoagulant drugs are often used clinically for cervical cancer patients to reduce the occurrence of VTE.

Enoxaparin sodium is mainly used for the prevention and treatment of various thromboembolic diseases. Its antithrombotic activity is comparable to that of heparin. Compared with other parenteral anticoagulants, it has rapid absorption and predictable pharmacokinetic characteristics. It has high bioavailability in vivo. It has a long half-life and low bleeding risk, can be administered by subcutaneous injection, and is more and more widely used in clinical practice [2]. However, affected by factors such as its pharmacological effect, injection method, and injection site selection, patients are prone to local pain, subcutaneous bleeding, and hematoma after subcutaneous injection.

Cervical cancer patients are at high risk of thrombosis, and the use of enoxaparin is high. Radiotherapy is one of the main treatment methods for cervical cancer, and 70% of cervical cancer patients require external pelvic irradiation. During pelvic radiotherapy, subcutaneous injection around the umbilicus is not feasible, and subcutaneous injection at the lower border of the deltoid muscle of the upper arm should be used instead. However, ecchymosis, hematoma, and even induration are prone to occur after injection at this site, which affects drug absorption, and the patient feels obvious pain. In addition to causing physical discomfort to patients, these symptoms can also have adverse psychological effects and limit subsequent injection sites [3]. There is a clinical study on the use of the abdominal imaginary line to make the injection positioning card and the symmetrical injection in the abdomen to reduce the subcutaneous hemorrhage caused by the low molecular weight heparin sodium injection [4]. However, subcutaneous injection at the lower margin of the upper arm deltoid muscle is the traditional injection method of the drug. Compared with abdominal injection, it is easier and faster and is more suitable for ambulatory patients. However, there is no study on the prevention of adverse events caused by subcutaneous injection of the upper arm deltoid muscle. Jinhuang Powder is prepared from turmeric, rhubarb, phellodendron, *Atractylodes*, *Magnolia officinalis*, dried tangerine peel, licorice, *Angelica*, and Trichosandra, which has repercussive and analgesic effects. In China, it is often used for carbuncle, furuncle, swelling and pain, traumatic injury, acute lymphadenitis, mastitis, and other diseases in clinics. The combination of these herbs has the effects of dispersing blood stasis and dredging collaterals, reducing swelling and analgesia, clearing heat, and dehumidifying. At present, Jinhuang Powder combined with honey, iced potato chips, and other related items has been used to treat subcutaneous hematoma caused by anticoagulant drugs or venipuncture [5, 6]. In this paper, the effect of Jinhuang Powder on the prevention and treatment of local complications after subcutaneous injection of enoxaparin sodium in the deltoid muscle of the upper arm is discussed retrospectively, and a new method is provided for clinical practice.

## 2. Materials and Methods

### 2.1. Research Subjects

The clinical data of cervical cancer patients who received pelvic external radiation and received enoxaparin sodium anticoagulation in our hospital from August 2020 to August 2021 were analyzed retrospectively. All patients received a subcutaneous injection of enoxaparin sodium through the lower border of the deltoid muscle of the upper arm. Patients were divided into two groups according to the use time of Jinhuang Powder: the research group was treated with topical Jinhuang Powder from the time of injection of enoxaparin sodium, and the control group was treated with topical Jinhuang Powder after subcutaneous induration, subcutaneous bleeding, or pain. This retrospective study complies with ethical requirements (ethical approval number: IRB-2020-276).

### 2.2. How to Use Jinhuang Powder

8 g of Jinhuang Powder was added to 10 ml of normal saline, and they are mixed well. The thickness of the application is 1.5–2 mm, and the range is 5 cm × 5 cm. We wrap it with a disposable treatment towel, avoid the puncture needle, and change the dressing every day. Research group: from the first day of injection of heparin sodium, every day after subcutaneous injection of enoxaparin sodium at the lower edge of the deltoid muscle of the upper arm for 30 minutes, the top of the puncture site was externally applied with Jinhuang Powder. Control group: after subcutaneous injection, only routine nursing was performed, and when pain, induration, or hematoma occurred, Jinhuang Powder was applied locally. The method was the same as that of the research group. The injection methods of enoxaparin sodium in the two groups were the same, and and kept for 5 s after the injection. The purpose was to wait for the basic diffusion of the drug solution and avoid excessive retention of the drug solution at the needle tip. The needle was withdrawn, and the needle plug was withdrawn at the same time to avoid leaving a small amount in the needle cavity. The liquid medicine is brought into the eye of the needle with the needle tip, irritating the skin and causing bleeding [7].

### 2.3. Observation Indicators and Evaluation Criteria [8]

The criteria are as follows: (1) the appearance and duration of subcutaneous induration; (2) subcutaneous hemorrhage: a hematoma with a diameter of less than 2 mm is called a bleeding point (Figure 1); a hematoma with a diameter of 3–5 mm or more, which does not fade under pressure, is called purpura (Figure 2); a hematoma with a diameter greater than 5 mm is called ecchymosis (Figure 3); those with a diameter greater than 10 mm, with local bulges or fluctuations, are called subcutaneous hematoma (Figure 4); (3) local pain score. It is divided into 5 grades. Grade 0 means that the patient does not feel pain; grade 1 means that the patient feels tenderness, but the patient can tolerate it without treatment; grade 2 means the degree of pain of the patient is very obvious; grade 3 is that the patient has severe tenderness and needs medical intervention; grade 4 is that the patient refuses any touch because of pain, and the degree of pain affects sleep.

## 3. Statistical Methods

Statistical analysis was performed using IBM SPSS v24. The *t*-test was used for measurement data that conformed to normal distribution, and chi-square analysis was used for count data. *P* < 0.05 was considered statistically significant.

## 4. Results

1. There were no significant differences in age, BMI, underlying diseases, ECO score, and coagulation indexes between the two groups. There were statistical differences in diabetes history and concurrent chemotherapy between the two groups. The characteristics of the two groups are shown in Table 1.
2. There were 2 cases of subcutaneous induration in the research group, the appearance time was 8.5 ± 0.7 days, and the duration was 5.5 ± 2.1 days; there were 6 cases of subcutaneous induration in the control group, and the appearance time was 8.2 ± 1.7 days and lasted for 8.5 ± 2.5 days. The incidence of induration in the research group was significantly lower than that in the control group (*P* < 0.05); the appearance time of induration was similar between the two groups, and there was no statistical significance; the duration of induration in the research group was less than that in the control group, but there was no significant difference (*P*=0.184) (Table 2).
3. The incidence of subcutaneous hemorrhage in the research group was significantly lower than that in the control group (37.9% vs 76.9%, *P*=0.003). In the research group, the appearance time of purpura, ecchymosis, and the hematoma was slightly delayed, and the duration was slightly shortened. The time of the appearance in the two groups was 6.1 ± 2.0 vs 6.0 ± 1.6, 6.3 ± 1.5 vs 7.6 ± 2.4, and 5.6 ± 2.4 vs 4.3 ± 1.3, and the duration was 8.4 ± 2.4 vs 9.8 ± 1.5, 8.3 ± 2.1 vs 11.2 ± 2.4, and 8.0 ± 3.4 vs 8.6 ± 2.6 days (Table 3).
4. The incidence of pain in the research group was significantly lower than that in the control group. The incidences of grade 0–4 pain in the two groups were 70% vs 28.2%, 19% vs 30.8%, 8.6% vs 23.1%, 1.7% vs 12.8%, and 1.7% vs 5.1%, respectively, with *P*=0.001. The time of onset of grade 2 and above pain was similar between the two groups, but the duration of pain was 4.7 ± 1.5 days in the research group and 9.6 ± 6.5 days in the control group. (Table 4).

## 5. Discussion

There is no clear plan for the prevention of side effects after subcutaneous injection of enoxaparin sodium in the arm deltoid muscle. This study compared the prophylactic and therapeutic use of topical Jinhuang Powder. The results showed that the preventive use of golden yellow powder could significantly reduce the incidence of sclerosis and subcutaneous hemorrhage caused by subcutaneous injection of enoxaparin sodium and effectively relieve local pain during injection.

Injection induration is due to the high concentration of the local drug and the hypertonic state, which is not easy to absorb, but absorbs the moisture of the surrounding tissue, causing local swelling. The outer edge of the deltoid muscle of the upper arm and the outer side of the thigh have a small injection range and a thin subcutaneous fat layer, which is not conducive to drug absorption, and repeated injections are prone to induration [9]. Traditional Chinese medicine believes that injection induration is caused by obstruction of the meridians, stagnation of qi, and blood stasis [10]. The ingredients of Jinhuang Powder include turmeric, rhubarb, phellodendron, *Atractylodes*, *Magnolia officinalis*, dried tangerine peel, licorice, Radix Radix, *Angelica dahurica*, and Trichosandra. Rhubarb has the effects of promoting blood circulation and eliminating blood stasis, clearing heat, and detoxifying. *Angelica dahurica* can warm and dispel wind and dry dampness, reduce swelling, and relieve pain. Modern pharmacological experiments have confirmed that phellodendron and turmeric can promote local blood circulation [11]. This study also found that the prophylactic use of Jinhuang Powder could not shorten the time of the formed subcutaneous induration, showing the importance of preventing the formation of induration. At the same time, after the formation of induration, it is necessary to find a more effective method to treat induration.

On the one hand, enoxaparin sodium is used due to its anticoagulant effect. After injection of the drug, the coagulation mechanism of the self-damaged capillaries is damaged and the coagulation time is prolonged. Compared with other drugs, subcutaneous bleeding events are more likely to occur after subcutaneous injection. On the other hand, the dermis is rich in capillaries, so when a patient is injected subcutaneously, local high concentrations of enoxaparin sodium may damage the blood vessels and cause local bleeding events [12]. So even after improving the injection method, the above situation still occurs. The phellodendron and turmeric in the Jinhuang Powder can promote local blood circulation and reduce vascular permeability. *Angelica* can reduce swelling and relieve pain. In addition, rhubarb in Jinhuang Powder can promote local vasoconstriction, shorten the bleeding time, and promote platelet adhesion and aggregation. In some studies, its hemostatic effect is even better than norepinephrine [13]. The results of this study show that the preventive use of Jinhuang Powder can significantly reduce the incidence of subcutaneous bleeding events caused by subcutaneous injection of enoxaparin sodium, which confirms the effect of Jinhuang Powder on reducing swelling and removing blood stasis. However, the prophylactic use of Jinhuang Powder did not cause subcutaneous bleeding events to subside faster than the therapeutic use of Jinhuang Powder. Therefore, prophylactic use should be emphasized in clinical use to reduce the occurrence of subcutaneous bleeding events.

Enoxaparin sodium can easily cause hematoma due to its subcutaneous injection. Once the hematoma is formed, the patient will show obvious pain, which not only brings pain to the patient but also makes it more difficult to continue subcutaneous injection in this area. Li et al. [11] have shown that the main chemical components of Jinhuang Powder are quercetin, *β*-sitosterol, stigmasterol, etc. Quercetin is a flavonoid compound that can effectively inhibit TNF (tumor necrosis factor) and IL (leukocyte). The expression of inflammatory factors such as interleukin) can dilate blood vessels and scavenge oxygen free radicals, thereby achieving anti-inflammatory, antioxidant, anti-inflammatory, and analgesic effects. A study has found that *β*-sitosterol has a strong anti-inflammatory effect on some nonspecific acute inflammations, and stigmasterol can significantly reduce IL-6 (interleukin 6), IL-1B (interleukin 1*β*), etc. [14]. The quercetin in the traditional Chinese medicine compound Jinhuangsan mainly comes from *Phellodendron phellodendri*, *β*-sitosterol mainly comes from *Phellodendron phellodendri*, rhubarb, and Tian Nanxing, and stigmasterol mainly comes from *Phellodendron phellodendri*, turmeric, and Tian Nanxing. Therefore, the combination of various drugs has a strong anti-inflammatory and analgesic effect, and the external application of Jinhuang Powder is also widely used in the treatment of phlebitis in clinics [15, 16]. Therefore, for patients with long anticoagulation courses, prophylactic use of Jinhuang Powder is beneficial to relieve pain and reduce the inflammatory response, which provides conditions for subsequent subcutaneous injections in this area.

In view of the side effects of subcutaneous injection of enoxaparin sodium, some scholars have studied the combination of Jinhuang Powder with other ingredients. Zhang [5] has shown that the use of Jinhuang Powder and honey modulation has a significant effect on subcutaneous induration caused by anticoagulant drugs. Xu [6] has shown that external application of iced potato chips can reduce tissue permeability, reduce exudation, and reduce swelling. Combined use with Jinhuang Powder can accelerate the absorption of hematoma. However, honey and iced potato chips are cumbersome in the process of storage and preparation and cannot guarantee sterility or cleanliness, which increases the risk of local infection. This study shows that the single use of Jinhuang Powder can not only reduce the workload but also achieve a good effect.

In conclusion, the prophylactic external application of Jinhuang Powder to patients who need a long-term subcutaneous injection of enoxaparin sodium can significantly reduce the incidence of subcutaneous induration and subcutaneous bleeding and can effectively relieve the local pain of injection. Further research is needed to clarify its role and mechanism. There are still deficiencies in this study. First, this study is a retrospective study, and the data are inevitably biased; second, the sample size of this study is small, and some phenomena cannot be explained at present, such as why the preventive use of Jinhuang Powder cannot shorten the formed induration and subcutaneous bleeding events; these need to be further studied.

## Figures and Tables

**Figure 1:** Bleeding point.

**Figure 2:** Purpura.

**Figure 3:** Ecchymosis.

**Figure 4:** Hematoma.

**Table 1:** Basic information of patients.

	Research group (*n* = 58)	Control group (*n* = 39)	*P*
Age (years)	60.2 ± 9.5	56.2 ± 10.7	0.056
BMI	23.19 ± 3.49	22.46 ± 3.67	0.328
Diabetes (*n*)			
Yes	9	0	0.010
No	49	39	
Hypertension (*n*)			
Yes	20	14	0.886
No	38	25	
ECO score (n)	1 (0–3)	1 (0–3)	0.224
Concurrent chemotherapy (*n*)			
Yes	38	35	0.007
No	20	4	
Platelet count (10/L)	239 ± 103	227 ± 119	0.600
Dimer (ng/ml)	1144.2 ± 1004.8	1070.7 ± 859.3	0.709
PT (s)	12.6 ± 1.2	12.8 ± 0.7	0.359
APTT(s)	29.1 ± 2.9	29.7 ± 3.7	0.342

**Table 2:** Cases of subcutaneous induration.

	Research group (*n* = 58)	Control group (*n* = 39)	*P*
Subcutaneous induration (*n*)	2	6	
No subcutaneous induration (*n*)	56	33	0.036
Time of occurrence (days)	8.5 ± 0.7	8.2 ± 1.7	0.807
Duration (days)	5.5 ± 2.1	8.5 ± 2.5	0.184

**Table 3:** Subcutaneous bleeding events.

	Research group (*n* = 58)	Control group (*n* = 39)	*P*
Grade of subcutaneous hemorrhage			0.003
No	36	9	
Bleeding point	7	13	
Purpura	7	5	
Ecchymosis	3	5	
Hematoma	5	7	
Occurrence time of purpura (days)	6.1 ± 2.0	6.0 ± 1.6	0.899
Purpura duration (days)	8.4 ± 2.4	9.8 ± 1.5	0.282
Occurrence time of ecchymosis (days)	6.3 ± 1.5	7.6 ± 2.4	0.452
Duration of ecchymosis (days)	8.3 ± 2.1	11.2 ± 2.4	0.137
Occurrence time of hematoma (days)	5.6 ± 2.4	4.3 ± 1.3	0.242
Duration of hematoma (days)	8.0 ± 3.4	8.6 ± 2.6	0.746

**Table 4:** Pain conditions.

	Research group (*n* = 58)	Control group (*n* = 39)	*P*
Pain grading			0.001
No	40	11	
Grade 1	11	12	
Grade 2	5	9	
Grade 3	1	5	
Grade 4	1	2	
Occurrence time of grade 2 and above pain (days)	6.7 ± 1.9	6.0 ± 2.3	0.481
Pain duration of grade 2 and above (days)	4.7 ± 1.5	9.6 ± 6.5	0.064

## Data Availability

The data used and/or analyzed during the current study are available from the corresponding author.

## References

[1] Trugilho I. D. A., Renni M. J. P., Medeiros G. C., Thuler L. C. S., Bergmann A. (2020). Incidence and factors associated with venous thromboembolism in women with gynecologic cancer. *Thrombosis Research*.

[2] Iqbal Z., Cohen M. (2011). Enoxaparin: a pharmacologic and clinical review. *Expert Opinion on Pharmacotherapy*.

[3] Şendir M., Büyükyılmaz F., Çelik Z., Taşköprü İ (2015). Comparison of 3 methods to prevent pain and bruising after subcutaneous heparin administration. *Clinical Nurse Specialist*.

[4] Wysokinski W. E., Houghton D. E., Casanegra A. I. (2019). Comparison of apixaban to rivaroxaban and enoxaparin in acute cancer-associated venous thromboembolism. *American Journal of Hematology*.

[5] Zhang L. (2017). Effect observation and nursing of Jinhuang powder and honey external application in the treatment of subcutaneous induration caused by low molecular weight heparin calcium. *China Health Care & Nutrition*.

[6] Xu B. (2015). Observation on the efficacy of external application of Jinhuang Powder in the treatment of infusion phlebitis. *Chinese Practical Medicine*.

[7] Spyropoulos A. C., Goldin M., Giannis D. (2021). Efficacy and safety of therapeutic-dose heparin vs standard prophylactic or intermediate-dose heparins for Thromboprophylaxis in high-risk hospitalized patients with COVID-19: the HEP-COVID randomized clinical Trial. *JAMA Internal Medicine*.

[8] Zhan H. B., Sun Q. Q., Yan L., Cai J. (2021). Clinical study of MEBO combined with jinhuang powder for diabetic foot with infection. *Evidence-based Complementary and Alternative Medicine*.

[9] Sun H., Ma X., Li Z., Liu J., Wang W., Qi X. (2021). Release characteristics of enoxaparin sodium-loaded polymethylmethacrylate bone cement. *Journal of Orthopaedic Surgery and Research*.

[10] Wu M., Huang J., Shi J., Shi L., Zeng Q., Wang H. (2022). Ruyi Jinhuang Powder accelerated diabetic ulcer wound healing by regulating Wnt/*β*-catenin signaling pathway of fibroblasts in Vivo and in Vitro. *Journal of Ethnopharmacology*.

[11] Li Q., Sun Y., Guo H. (2018). Quality control of the traditional Chinese medicine Ruyi jinhuang powder based on high-throughput sequencing and real-time PCR. *Scientific Reports*.

[12] Yeh Y. C., Wang M. J., Lin C. P. (2012). Enoxaparin sodium prevents intestinal microcirculatory dysfunction in endotoxemic rats. *Critical Care*.

[13] Liu J. T., Wu J., Wang H. R. (2020). Spraying rhubarb powder solution under gastroscope in the treatment of acute non-varicose upper gastrointestinal bleeding: a systematic review and meta-analysis of randomized controlled trials. *Complementary Therapies in Medicine*.

[14] Paniagua-Pérez R., Flores-Mondragón G., Reyes-Legorreta C. (2016). Evaluation of the anti-inflammatory capacity of beta-sitosterol in rodent assays. *African Journal of Traditional, Complementary and Alternative Medicines*.

[15] Ahmad Khan M., Sarwar A. H. M. G., Rahat R., Ahmed R. S., Umar S. (2020). Stigmasterol protects rats from collagen induced arthritis by inhibiting proinflammatory cytokines. *International Immunopharmacology*.

[16] Zeng M., Liao Q., Cui Y., Tang H., Yu M. (2021). The therapeutic efficacy and safety of traditional Chinese medicine injection combined with low-molecular-weight heparin on the acute lower extremity deep venous thrombosis: a protocol for systematic review and network meta-analysis. *Medicine (Baltimore)*.

